The article "MicroR‐9‐5p suppresses EV71 replication through targeting NFκB of the RIG‐I‐mediated innate immune response" was retracted in 2023. Reasons: duplicate publication; signs of a paper mill; unreliable results or conclusions.

# MicroR‐9‐5p suppresses EV71 replication through targeting NFκB of the RIG‐I‐mediated innate immune response

**DOI:** 10.1002/2211-5463.12490

**Published:** 2018-08-29

**Authors:** Bing Li, Junqing Zheng

**Affiliations:** ^1^ Department of Pediatrics Jinan Maternity and Child Care Hospital China

**Keywords:** EV71, inflammation, innate immunity, miR‐9, NFκB

## Abstract

Accumulating evidence demonstrates that there is a causative link between hsa‐microRNA‐9‐5p (miR‐9) and pathophysiological processes. Enterovirus 71 (EV71) has been found to contribute to numerous severe clinical symptoms which result in death. The exact mechanism by which EV71 influences miR‐9 expression is unknown, and the relationship between miR‐9 and EV71 is still unclear. Here, miR‐9 expression was found to be impaired upon EV71 infection in several cell lines and in an EV71 infection mouse model. Additionally, we confirmed that EV71 infection induces robust expression of pro‐inflammatory cytokines (TNF‐α, IL‐6, and IL‐1) and interferons (IFN‐α and IFN‐β). Overexpression of miR‐9 attenuated EV71 proliferation and reduced protein and gene expressions of virion protein 1 (VP1) of EV71. Furthermore, we observed that the inflammation caused by EV71 infection was restored to a moderate level via miR‐9 overexpression. Nuclear factor kappa B (NFκB) in the retinoic acid‐induced gene 1 (RIG‐I) signaling pathway, but not interferon regulating factor 3 (IRF3), was significantly decreased and inactivated by ectopic miR‐9 expression. Moreover, in mouse infection experiments, administration of miR‐9 agomirs caused a significant decrease in VP1 levels and pro‐inflammatory cytokine production after viral inoculation. Taken together, the present data demonstrate that miR‐9 exerts an anti‐EV71 effect in cells and a mouse model via mediating NFκB activity of the RIG‐I signal pathway, thereby suggesting a new candidate for antiviral drug development.

**Abbreviations**
BSA: bovine serum albumin
CARD: caspase‐recruitment domain
DMEM: Dulbecco's modified Eagle's medium
EV71: enterovirus 71
FBS: fetal bovine serum
HEK: human embryonic kidney
HFMD: hand, foot, and mouth disease
IL: interleukin
IRF3: interferon regulating factor 3
miR‐9: hsa‐microRNA‐9‐5p
MOI: multiplicity of infection
NFκB: nuclear factor kappa B
PAMPs: pathogen‐associated molecular patterns
PRR: pattern recognition receptor
RIG‐I: retinoic acid‐induced gene 1
RLR: RIG‐I‐like receptor
TLR: Toll‐like receptor
TNF‐α: tumor necrosis factor‐alpha
VP1: virion protein 1

Hand, foot, and mouth disease (HFMD) is a viral infection commonly occurring in children and infants, which produces flu‐like symptoms and blisters 1, 2, 3. HFMD is caused by enteroviruses [e.g., coxsackievirus A16 and enterovirus 71 (EV71)] 4, 5, 6. EV71 is a single‐stranded positive‐sense RNA virus belonging to the *Enterovirus* genus of the Picornaviridae family 7, 8. Infection by EV71 in children is related to severe neurological, pulmonary, and gastrointestinal dysfunctions. It has been suggested that disease severity is additionally affected by host factors, such as the host immune response 9. The severity of EV71 infection has been found to be related to excessive and robust pro‐inflammatory chemokine and cytokine responses and production 10.

The article "MicroR‐9‐5p suppresses EV71 replication through targeting NFκB of the RIG‐I‐mediated innate immune response" was retracted in 2023. Reasons: duplicate publication; signs of a paper mill; unreliable results or conclusions.

The innate immune system affords defense against invading pathogens at an early phase of infection by recognizing various conserved pathogen‐associated molecular patterns (PAMPs), including viral RNAs, and acting to limit virus replication. RLRs (RIG‐I‐like receptors) 11, TLRs (Toll‐like receptors) 12, and NOD‐like receptors 13 are members of PRRs (pattern recognition receptors), which can recognize viral RNA and elicit downstream signal transduction to provoke the innate immune response. Innate immunity is utilized by the host to fight against foreign pathogens, and EV71 invasion triggers the RLR and TLR pathways to counter the duplication and spreading of the virus. RIG‐I, an essential receptor that recognizes EV71 RNA, engages in cytokine production in the host. RIG‐I releases the N‐terminal caspase‐recruitment domain (CARD) for interaction with an identical domain on the adaptor protein located on the outer membrane of mitochondria after it interacts with viral RNAs 14, and consequently activates nuclear factor kappa B (NFκB) and interferon regulating factor 3/7 (IRF3/7). Phosphorylation of NFκB and IRF3/7 induces production of pro‐inflammatory cytokines, chemokines, interferon (IFN), and adhesion molecules against pathogen invasion. However, the hyperinduction of pro‐inflammatory cytokines induced by pathogen infection, such as tumor necrosis factor (TNF)‐α, interleukin (IL)‐1, and IL‐6 (i.e., a cytokine storm), causes complications or even ultimately death as a result of these infections 15.

The microRNAs (miRs) belong to a group of small noncoding RNAs, which were first identified in *C. elegans* in 1993 16. Previous reports demonstrated that miRs function in many pathological and biological processes, including inflammation and viral infection 17, 18, 19, 20, 21, 22. MicroRNAs additionally play an essential role in EV71 infection and modulating viral replication and pathogenicity 23, 24, 25. In our study, we found that EV71 infection downregulated the expression of miR‐9. Ectopic expression of miR‐9 with EV71 infection induced an RLR‐triggered innate immune response and pro‐inflammatory cytokine production. Moreover, miR‐9 agomirs were able to limit EV71 replication by maintaining cytokines at a moderate level in different tissues in animal model. Notably, our data reveal that miR‐9 significantly decreased EV71‐induced excessive production of pro‐inflammatory cytokines through reducing expression and activation of NFκB. Given these results, our data demonstrate that miR‐9 positively regulates inflammation elicited by EV71 and suppresses virus replication by targeting NFκB.

The article "MicroR‐9‐5p suppresses EV71 replication through targeting NFκB of the RIG‐I‐mediated innate immune response" was retracted in 2023. Reasons: duplicate publication; signs of a paper mill; unreliable results or conclusions.

## Materials and methods

### Cell culture

Human embryonic kidney (HEK) 293T cells, human rhabdomyosarcoma cells (RD), human cervical carcinoma cells (HeLa), human colorectal cells (HT‐29), Vero cells, and human monocytes (THP‐1) were obtained from ATCC (Manassas, VA, USA) and maintained in Dulbecco's modified Eagle's medium (DMEM; Gibco, Shanghai, China) supplemented with 2% penicillin/streptomycin and 10% (v/v) fetal bovine serum (FBS; Gibco) at 5% CO_2_ and 37 °C. This work was approved by Jinan Maternity and Child Care Hospital.

### Virus propagation

Enterovirus 71 (Shenzhen strain, GenBank accession number AF30299.1) infection was performed as follows. Vero cells were used to produce human EV71. Briefly, Vero cells were seeded into a dish prior to infection. EV71 was dispersed in DMEM, followed by inoculation to Vero cells (approximately 80% confluence). We added DMEM supplemented with 2% FBS, and the infection was allowed to proceed until the monolayer showed cytopathic effects (CPE). The culture medium and cells were harvested and subjected to three freeze‐thaw cycles. Ten‐minute centrifugation at 4500 ***g*** was performed, and the supernatant was transferred into cryovials and stored at −80 °C.

### The 50% tissue culture infectious dose titration

The 50% tissue culture infectious dose (TCID_50_)/mL titration was determined for the virus as follows. Briefly, we seeded ~5000 RD cells/well in a 96‐well plate. DMEM supplemented with FBS (2%; 10^3^ to 10^8^ dilution) was used to dilute the virus, and each dilution was added in separate wells. The plates underwent incubation at 5% CO_2_ and 37 °C for 2 to 5 days. Using microscopy, CPE was analyzed. Reed–Münch endpoint calculation was employed to determine TCID_50_.

### EV71 infection

Enterovirus 71 infection of 293T, Vero, RD, HT‐29, HeLa, and THP‐1 cells was performed. Specifically, EV71 was inoculated into monolayer cells at approximately 50% confluence at a multiplicity of infection (MOI) of 1–10 TCID_50_/cell. After 1 h of adsorption in an incubator at 37 °C and 5% CO_2_, culture medium without FBS was used to wash the cells to remove free virus. Then, fresh culture medium supplemented with FBS (10%) was added. Cells were harvested for further examination at the indicated time points.

The article "MicroR‐9‐5p suppresses EV71 replication through targeting NFκB of the RIG‐I‐mediated innate immune response" was retracted in 2023. Reasons: duplicate publication; signs of a paper mill; unreliable results or conclusions.

### Animal infection models

Pregnant mice (ICR) were provided by Vital River (Beijing, China). All of the mice were raised in a pathogen‐free room with separate ventilation cage systems. The mice were aged for two weeks and then were infected with either sterile PBS or EV71 at the dose of 10^5^ TCID_50_/mouse via an intraperitoneal route. Disease manifestations and weight were observed and recorded every day following infection. The animals were sacrificed four or five days after posterior paralysis appeared. Muscle tissue, spleen, heart, lung, brain, kidney, small intestine, and whole blood were harvested, and RNA was extracted.

All experiments followed the institutional guidelines for animal research, and approval was obtained from the Ethics Committee of the Jinan Maternity and Child Care Hospital.

### Antibodies

Anti‐VP1 (from Shenzhen strain, bs‐2297R), monoclonal anti‐β‐actin (ab8227), anti‐RIG‐I (sc‐376845), anti‐IL‐1 (ab9722), anti‐IFN‐β (ab151605), and anti‐NFκB (ab16502), anti‐IRF3 (ab25950), anti‐phospho‐NFκB (ab86299), and anti‐phospho‐IRF3 (ab192796) antibodies were purchased from Abcam (CA, USA) and Santa Cruz Biotechnology, Inc. (Santa Cruz, CA, USA) to detect the indicated protein by western blotting. Goat anti‐rabbit IgG conjugated to TRITC (tetramethyl rhodamine isothiocyanate) secondary antibodies was purchased from Zhongshan Golden Bridge Biotechnology (Beijing, China) and was used for immunofluorescence assay (IFA).

### Western blotting

Cells were lysed in RIPA buffer (pH 8.0, 50 mm Tris/HCl, 150 mm NaCl, 1% NP‐40, 0.1% SDS) containing a protease inhibitor cocktail. The BCA Protein Quantitation Kit was used to determine the protein concentration. SDS/PAGE (10%) was used to separate protein samples (20 μL, 1 mg·mL^−1^), which were then electrically transferred onto Immobilon PVDF membranes (0.45 μm). The membranes were then blocked with BSA (bovine serum albumin; 5%) in PBST (0.5% Triton X‐100 added in PBS) at room temperature for 1 h, followed by overnight incubation at 4 °C with the following antibodies: rabbit anti‐VP1 (1 : 2500), anti‐RIG‐I (1 : 5000), anti‐IRF3 (1 : 1000), mouse anti‐phospho‐IRF3 (1 : 500), anti‐NFκB (1 : 2000), anti‐phospho‐NFκB (1 : 500), and anti‐β‐actin (1 : 2500). Then, Amersham ECL peroxidase‐linked goat anti‐mouse IgG or anti‐rabbit IgG secondary antibodies were incubated with the membranes for 1 h at 25 °C. The C‐DiGit Blot Scanner and SuperSignal West Femto Maximum Sensitivity Substrate Kit (Thermo Fisher Scientific, Waltham, MA, USA) were used to detect western blot immunoreactivity.

The article "MicroR‐9‐5p suppresses EV71 replication through targeting NFκB of the RIG‐I‐mediated innate immune response" was retracted in 2023. Reasons: duplicate publication; signs of a paper mill; unreliable results or conclusions.

### RNA extraction and real‐time PCR

Total RNA was extracted from the cells after the indicated treatments using TRIzol reagent (Invitrogen, Carlsbad, CA, USA) according to the manufacturer's instructions. The levels of mRNA were determined using SYBR Green Master Mix (4385618; Thermo Fisher Scientific) incorporation on a Roche LightCycler 480 Real‐Time PCR system (Roche, Basel, Switzerland), and GAPDH was used as the internal control. The sequences of the primers used are shown in Table 1.

**Table 1:** Primer sequences

Full name	Abbreviation
miR‐9 F	5′‐GGT CTT TGG TTA TCT AGC TGT ATG A‐3′
miR‐9 R	5′‐GTG CAG GGT CCG AGG T‐3′
VP1 F	5′‐GCT CTA TAG GAG ATA GTG TGA GTA GGG‐3′
VP1 R	5′‐ATG ACT GCT CAC CTG CGT GTT‐3′
RIG‐I F	5′‐GGA CGT GGC AAA ACA AAT CAG‐3′
RIG‐I R	5′‐GCA ATG TCA ATG CCT TCA TCA‐3′
Human IL‐1 F	5′‐TGA AAT GCC ACC TTT TGA CAG‐3′
Human IL‐1 R	5′‐CCA CAG CCA CAA TGA GTG ATA C‐3′
Mouse IL‐1 F	5′‐GCA CTA CAG GCT CCG AGA TGA AC‐3′
Mouse IL‐1 R	5′‐TTG TCG TTG CTT GGT TCT CCT TGT‐3′
IL‐6 F	5′‐TGC CTT CTT GGG ACT GAT‐3′
IL‐6 R:	5′‐CTG GCT TTG TCT TTC TTG TT‐3′
TNF‐α F	5′‐CGA TGA GGT CAA TCT GCC CA‐3′
TNF‐α R	5′‐CCA GGT CAC TGT CCC AGC‐3′
IFN‐α F	5′‐TAA TTC CTA CGT CTT TTC TTT‐3′
IFN‐α R	5′‐TAT GCC TGA TCC CTG AAC AGT‐3′
Human IFN‐β F	5′‐TAG CAC TGG CTG GAA TGA GA‐3′
Human IFN‐β R	5′‐TCC TTG GCC TTC AGG TAA T‐3′
Mouse IFN‐β F	5′‐AAG AGT TAC ACT GCC TTT GCC ATC‐3′
Mouse IFN‐β R	5′‐CAC TGT CTG CTG GTG GAG TTC ATC‐3′
GAPDH F	5′‐GGA AAG CTG TGG CGT GAT‐3′
GAPDH R	5′‐AAG GTG GAA GAA TGG GAG TT‐3′

Quantitative real‐time PCR was performed in 20 μL volumes using the SYBR Green PCR Master Mix in the LightCycler 480 with the following conditions: 95 °C for 10 min, then 40 cycles of 95 °C for 15 s, 60 °C for 30 s, and 72 °C for 30 s. The level of each mRNA (2^−ΔΔCT^) was calculated through normalization to the endogenous reference and relative to the calibrator (the mean of the control samples).

### Immunofluorescence assays

Virus infection of RD cells grown in 24‐well plates with cover slides was performed at an MOI of 0.1 TCID_50_/cell. Paraformaldehyde (4%) in PBS was used to fix the cells for 1 h at room temperature. Ten‐minute permeabilization of the cells with PBST was performed at 25 °C, followed by a 1‐h incubation with PBST (including 0.4% BSA) at 37 °C and a subsequent 1‐h incubation with polyclonal anti‐VP1 antibody, which was diluted in PBST (including 0.2% BSA) at 37 °C. Following a 1‐h PBST wash, the cells underwent 1‐h incubation with TRITC‐labeled goat anti‐rabbit antibody diluted in 0.2% BSA and PBST at 37 °C. Next, cells were washed for 1 h with PBST. DAPI was used to stain the nuclei of the cells. A confocal laser scanning fluorescence microscope (Olympus LSCMFV500, Olympus, Tokyo, Japan) was employed to analyze VP1 staining in cells.

The article "MicroR‐9‐5p suppresses EV71 replication through targeting NFκB of the RIG‐I‐mediated innate immune response" was retracted in 2023. Reasons: duplicate publication; signs of a paper mill; unreliable results or conclusions.

### miR‐9‐mimic and miR‐9 agomir preparation

miR‐9‐mimic and a scramble control, NC‐mimic, were purchased from Genscript (Shanghai, China). miR‐9‐mimic is an artificial, chemically modified double‐stranded miRNA, which mimics the mature endogenous miR‐9 after being transfected into cells with concentration of 100 μg·mL^−1^. Both miR‐9‐mimic and NC‐mimic were suspended in 0.9% NaCl to a final storage concentration of 10 mg·mL^−1^.

The miR‐9 agomir is a double‐stranded RNA analog of mature miR‐9 which has been chemically modified and conjugated to a cholesterol moiety to promote specificity and stability for assays. For treatment *in vivo*, agomiR‐9 (RiboBio, Guangdong, China) was injected intravenously into the tail vein at a dose of 1 nmol (diluted in 20 μL PBS) per mouse three days before EV71 infection.

### Bioinformatics analysis

The potential targets of miR‐9 were identified by combining algorithms using miRDB (http://www.mirdb.org). The targets predicted by these algorithms were analyzed, and the candidates were selected according to the function.

### Dual‐luciferase reporter assay

Amplification of the 3′‐UTR of the NFκB gene was performed, which was inserted into the GV126 luciferase gene. The binding sites for miR‐9 on the NFκB gene were destroyed by mutagenesis, and the mutants were selected as controls. The transfection efficiency was adjusted by the thymidine kinase promoter (pRL‐TK vector; TaKaRa, Beijing, China) and the Renilla luciferase gene, which contained the plasmid. Cotransfection of miR‐9‐mimic and NC‐mimic into the luciferase reporter vector was conducted for different cell lines with Lipo2000 transfection reagent. The luciferase assay was performed according to the manufacturer's instructions. Myllicin (to avoid any possibility of the fungal and/or bacterial infection during handling the experiments) was added into the cell culture in DMEM (supplemented with 10% FBS), followed by incubation at 5% CO_2_ and 37 °C. The medium was changed every two days. Then, 0.25% trypsin was used to detach the cells, followed by subculture when the cells reached ~70–80% confluency.

### Statistical analysis

The data are presented as the mean ± standard deviation. Two‐tailed Student's t‐test was employed for comparison. Values of *P* < 0.05 were considered statistically significant: *P < 0.05; **P < 0.01; and ***P < 0.001.

## Results

### miR‐9 expression decreases during EV71 infection

The miR‐9 expression in 293T, Vero, RD, HT‐29, HeLa, and THP‐1 cells was examined at 24 h after EV71 infection. Virion protein 1 (VP1) expression was found to be markedly increased in each of these six cell lines after EV71 infection at both the protein and mRNA levels (Fig. 1A,B), indicating the successful infection by EV71. We then found that miR‐9 expression was significant decreased after EV71 infection in all cell lines, especially in RD cells. Next, EV71‐infected mice were utilized to examine miR‐9 expression *in vivo*. The EV71 was injected into the abdomen of the mice, which were sacrificed either four or five days following appearance of severe posterior paralysis. Real‐time PCR analysis revealed that the virus mainly localized to the lung and muscle (Fig. 1C). There were relatively low titers of EV71 in the spleen, brain, liver, and intestine. The expression level of miR‐9 in different tissues was then examined. We observed a significant decrease in miR‐9 expression in muscle, intestine, lung, and brain (Fig. 1D). Taken together, these data demonstrate that EV71 mainly replicates in muscle. The downregulation of miR‐9 in muscle induced by EV71 infection was verified by real‐time PCR (Fig. 1E).

The article "MicroR‐9‐5p suppresses EV71 replication through targeting NFκB of the RIG‐I‐mediated innate immune response" was retracted in 2023. Reasons: duplicate publication; signs of a paper mill; unreliable results or conclusions.

**Figure 1:** miR‐9 expression level in EV71‐infected cells and mice. (A and B) Increased expression of VP1 at the protein and mRNA levels in EV71‐infected cell lines was observed compared to noninfected cells (NC). (C) A reduced expression level of miR‐9 was observed in EV71‐infected cell lines compared with the negative control. (D and E) Expression level of VP1 and miR‐9 in different tissues of EV71‐infected and noninfected mice was examined using real‐time PCR. These assays have been performed three times. Data represent means ± SD. *P < 0.05; **P < 0.01; ***P < 0.001. The statistical test performed using Student's *t*‐test.

### EV71 infection causes pro‐inflammatory cytokine production

To confirm whether EV71 infection causes robust production of pro‐inflammatory cytokines, real‐time PCR and western blotting were conducted to assess the expression of IL‐1, IL‐6, TNF‐α, IFN‐β, and IFN‐α at the protein and mRNA levels after EV71 infection of human colorectal, Vero, and rhabdomyosarcoma cells. As Fig. 2A shows, IL‐1 and IFN‐β expression in three cell lines was significantly increased in the EV71‐infected group. Real‐time PCR data further confirmed that IL‐1, IL‐6, TNF‐α, IFN‐α, and IFN‐β mRNA levels were significantly elevated after EV71 infection, especially in RD cells (Fig. 2B). Next, the EV71‐infected mouse model was utilized to evaluate relative IL‐1 and IFN‐α expression in several tissues. As expected, excessive production of cytokines was observed in muscle and lung tissue (Fig. 2C). These data clearly demonstrate that EV71 invasion induces pro‐inflammatory cytokine production *in vitro* and *in vivo*.

The article "MicroR‐9‐5p suppresses EV71 replication through targeting NFκB of the RIG‐I‐mediated innate immune response" was retracted in 2023. Reasons: duplicate publication; signs of a paper mill; unreliable results or conclusions.

**Figure 2:** EV71 infection shows a stimulatory effect on pro‐inflammatory cytokine production in cells and in an animal model. Human colorectal cells, Vero, and rhabdomyosarcoma cells were infected with EV71 for 8 h. The expressions of pro‐inflammatory cytokines IL‐1, IL‐6, TNF‐α, IFN‐α, and IFN‐β of infected cells were examined by western blotting (A) and real‐time PCR (B) at the indicated time points. (C) Mice from the EV71 group and the NC group were sacrificed on day 4 or 5 postinoculation to determine the expressions of IL‐1 and IFN‐β in different tissues of mice. These assays have been performed three times. Data represent means ± SD. *P < 0.05; **P < 0.01; ***P < 0.001. The statistical test performed using Student's *t*‐test.

### Ectopic expression of miR‐9 inhibits EV71 replication

After human colorectal, Vero, and rhabdomyosarcoma cells were infected with EV71 and/or transfected with miR‐9‐mimic, multiple growth curves were determined to assess the influence of miR‐9 on EV71 replication. As shown in Fig. 3A, the viral growth rate was significantly reduced by 10^2^‐ to 10^5^‐fold in miR‐9‐mimic‐treated cells. The virion protein 1 (VP1) was examined at the protein and mRNA levels at the indicated time points. As shown in Fig. 3B, VP1 expression was significantly decreased by miR‐9‐mimic transfection, especially in RD cells, in which its expression pattern was markedly reduced. The decrease in viral protein was consistent with real‐time PCR results, which showed that the mRNA level of VP1 was significantly reduced in the miR‐9‐mimic‐treated group compared with the nontreated group (Fig. 3C). We then performed IFA to visualize the VP1 in the infected RD cells. As shown in Fig. 3D, the level of VP1 in EV71‐infected cells treated with miR‐9‐mimic was significantly less than that in the nontreated group. These results suggest that miR‐9 significantly decreased the viral titers of EV71 in different cell lines.

**Figure 3:** miR‐9 attenuates the replication of EV71 replication. Vero, RD, and HT‐29 cells were infected with EV71. (A) At the indicated time points, titers of the viruses in the culture supernatants were determined in Vero, RD, and HT‐29 cells. Error bars represent the standard error of the mean from replicate samples. (B) The viral VP1 protein of EV71 was detected by western blotting at several time points during the first viral replication cycle (12, 24, and 36 h) in HT‐29, Vero, and RD cells. (C) Real‐time PCR was performed to detect VP1 expression of EV71 at different time points. (D) VP1 subcellular localization was examined by IFA after miR‐9‐mimic transfection and EV71 infection for 12 and 24 h. These assays have been performed three times. Data represent means ± SD. **P < 0.01. The statistical test performed using Student's *t*‐test.

The article "MicroR‐9‐5p suppresses EV71 replication through targeting NFκB of the RIG‐I‐mediated innate immune response" was retracted in 2023. Reasons: duplicate publication; signs of a paper mill; unreliable results or conclusions.

### miR‐9 inhibits excessive production of pro‐inflammatory cytokines induced by EV71

To confirm the effect of miR‐9 on pro‐inflammatory cytokine production at the cellular level, real‐time PCR was performed to evaluate the level of cytokines and interferon. Importantly, we found that three essential cytokines in EV71‐infected cells, IL‐1, IL‐6, and TNF‐α, were gradually induced at different stages of infectious cycle. However, their expressions were kept at a moderate level at the examined time points postinfection in the miR‐9‐mimic‐treated group (Fig. 4A). Furthermore, these cytokines in RD cells were examined by western blotting. In the EV71‐infected group, cytokine expression significantly increased, but their production was clearly suppressed by miR‐9 expression (Fig. 4B). These results indicate that miR‐9 ameliorated the robust cytokine storm induced by EV71 at the later stage of infection.

**Figure 4:** miR‐9‐mimic transfection suppresses pro‐inflammatory cytokine production in EV71‐infected cells. RD cells were transfected with miR‐9‐mimic and then infected with EV71 at 24 h postinfection. The expression of pro‐inflammatory cytokines IL‐1, IL‐6, TNF‐α, IFN‐α, and IFN‐β of infected cells was examined by (A) real‐time PCR and (B) western blotting at several time points. These assays have been performed three times. Data represent means ± SD. *P < 0.05; **P < 0.01; ***P < 0.001. The statistical test performed using Student's *t*‐test.

Enterovirus 71 viral infection can induce multiple innate immune signaling pathways, especially the RIG‐I‐like receptor (RLR) pathway. To determine whether the RIG‐I pathway plays an essential role in the miR‐9‐regulated host innate immune response to EV71 infection, analysis of RIG‐I and two key sensors (IRF3 and NFκB) was performed at the transcriptional and translational levels after EV71 infection and/or miR‐9‐mimic treatment (Fig. 5A). Protein expression of both IRF3 and RIG‐I in miR‐9‐mimic‐expressing cells did not show a significant difference with nontransfected cells. However, NFκB expression decreased after miR‐9‐mimic transfection compared to cells only induced by EV71. Additionally, phosphorylated NFκB, which is an indication of activated NFκB, was reduced, but phosphorylated IRF3 was not. Consistent with these results, real‐time PCR data suggested more efficient downregulation of NFκB was observed in RD cells treated with miR‐9‐mimic, while lower NFκB was detected in the miR‐9‐mimic‐treated group, compared to the nontreated group (Fig. 5B). Together, these data demonstrate that miR‐9 regulates inflammation production via the RIG‐I signal pathway.

The article "MicroR‐9‐5p suppresses EV71 replication through targeting NFκB of the RIG‐I‐mediated innate immune response" was retracted in 2023. Reasons: duplicate publication; signs of a paper mill; unreliable results or conclusions.

**Figure 5:** Activation of RIG‐I signal pathway is inhibited by miR‐9‐mimic transfection. RD cells were transfected with miR‐9‐mimic and then infected with EV71 at 24 h posttransfection. (A) Expression of RIG‐I, NFκB, phosphorylated NFκB, IRF3, and phosphorylated IRF3 of infected cells was examined by western blotting at several time points postinfection. (B) We performed real‐time PCR to examine gene expression of NFκB, RIG‐I, and IRF3 at several time points following infection. These assays have been performed three times. Data represent means ± SD. *P < 0.05; ***P < 0.001. The statistical test performed using Student's *t*‐test.

### NFκB is a target of miR‐9

Bioinformatics analysis has identified NFκB, which is a key immune sensor for the RLR innate immune response against EV71 infection, as a functional putative miR‐9 target (Fig. 6A). A dual‐luciferase reporter assay was conducted in six cell lines (293T, Vero, RD, HT‐29, HeLa, and THP‐1) to investigate direct binding between NFκB and miR‐9. The data show that miR‐9‐mimic transfection decreased the luciferase activity of the reported fused with the NFκB 3′‐UTR (Fig. 6B). Furthermore, we examined the NFκB expression in the six cell lines infected with EV71 and/or transfected with miR‐9‐mimic, using real‐time PCR and western blotting. As shown in Fig. 6C,D, the NFκB expression was suppressed because of miR‐9‐mimic expression at both the protein and mRNA levels.

**Figure 6:** NFκB is a direct target of miR‐9. (A) Graphical representation of the conserved miR‐9 binding motif in the 3′‐UTR of NFκB. The complementary sequences to the seed regions of miR‐9 and the corresponding sequence of 3′‐UTR of NFκB are conserved among three species. (B) The luciferase activity of the luciferase reporter constructs containing either the wild‐type or mutated 3′‐UTR of human NFκB after miR‐9‐mimic transfection in several cell lines. The luciferase activity was normalized to the activity of β‐galactosidase. miR‐9 overexpression significantly decreased the relative luciferase activity in the wild‐type 3′‐UTR, but not mutant 3′‐UTR of NFκB mRNA. (C and D) Western blotting and real‐time PCR analysis were performed to determine the levels of NFκB protein and mRNA after miR‐9‐mimic transfection or control. These assays have been performed three times. Data represent means ± SD. *P < 0.05; **P < 0.01; ***P < 0.001. The statistical test performed using Student's *t*‐test.

### miR‐9 agomir administration ameliorates the EV71‐induced inflammatory cytokine storm

To further probe the mechanism of how miR‐9 agomir administration attenuates EV71 replication and pathogenicity in an animal model, we performed real‐time PCR to assess VP1 and cytokine levels. As shown in Fig. 7A, miR‐9 was confirmed to be ectopically expressed by real‐time PCR. Additionally, we found that VP1 expression was significantly reduced after miR‐9 agomir administration, suggesting an antiviral effect of miR‐9. Furthermore, the levels of the pro‐inflammatory cytokines induced by EV71 were evaluated by real‐time PCR experiment (Fig. 7B). As shown in Fig. 7C,D, robust expression of IL‐1 and IFN‐β was observed in muscle, lung, blood, and spleen tissues of EV71‐infected mice. In contrast, the expression of these two cytokines was markedly inhibited with agomiR‐9 treatment. Together, our data provide evidence that miR‐9 confers an inhibitory effect on the EV71‐induced cytokine storm and therefore ameliorates the damage caused by EV71.

The article "MicroR‐9‐5p suppresses EV71 replication through targeting NFκB of the RIG‐I‐mediated innate immune response" was retracted in 2023. Reasons: duplicate publication; signs of a paper mill; unreliable results or conclusions.

**Figure 7:** Effect of miR‐9 on EV71 replication and pathogenicity in mice. Mice were inoculated with EV71 or PBS as a negative control. Mice were then treated with miR‐9 agomir. (A) Mice from the EV71 group and the NC group were sacrificed on day 4 or 5 postinoculation to determine miR‐9 expression in different tissues of mice. Expression levels of VP1 (B), IL‐1 (C), and IFN‐β (D) in different tissues of EV71‐infected mice were examined using real‐time PCR. These assays have been performed three times. Data represent means ± SD. *P < 0.05; **P < 0.01; ***P < 0.001. The statistical test performed using Student's *t*‐test.

## Discussion

In this study, an inhibitory role of miR‐9 in replication and pathogenicity of EV71 infection was observed both *in vitro* and *in vivo*. The expression pattern of viral EV71 protein was decreased by miR‐9 treatment. Furthermore, we found that miR‐9 was able to ameliorate the robust innate immune response against EV71 at different stages of infection by targeting the immune sensor NFκB and decreasing its expression.

Increasing evidence has demonstrated that excessive inflammatory signaling occurring during organ injury is one of the main pathogenic factors responsible for high mortality following EV71 infection 26, 27, 28. NFκB is a signaling pathway that regulates many genes related to cell differentiation, proliferation, and innate immune response. In addition, via eliciting pro‐inflammatory cytokine and type I IFN (IFN‐β and IFN‐α) expression, NFκB is important in the antiviral reactions of the host 29, 30, 31. However, the 2C protein of EV71 suppresses NFκB activation, which increases the virus replication. Viral protein 2C suppresses the phosphorylation of IκBα and IKKβ via binding with their kinase domains, reducing NFκB activation, and promoting viral replication 32. In our study, miR‐9 administration resulted in deactivation and expression of NFκB while inhibiting EV71 replication. These results could be attributed to the robust pro‐inflammatory cytokines, which are believed to contribute to EV71 pathogenicity, which were ameliorated by miR‐9 expression, indicating that a moderate level of cytokines and interferon was maintained to limit the effect of EV71. However, the molecular mechanisms by which miR‐9 controls VP1 expression and viral replication during EV71 infection still need further research to investigate the possibility of whether miR‐9 inhibits inflammation and EV71 propagation separately.

The article "MicroR‐9‐5p suppresses EV71 replication through targeting NFκB of the RIG‐I‐mediated innate immune response" was retracted in 2023. Reasons: duplicate publication; signs of a paper mill; unreliable results or conclusions.

The practical implication of miR‐9 in evolution is suggested by its sequence conservation at the nucleotide level in different species rather than its varying expression patterns. Although the sequence of miR‐9 is conserved, its expression profile differs significantly in various species. miR‐9 is being extensively investigated in various biological processes: NPC proliferation and migration 33, neuronal differentiation 34, apoptotic cell death 35, brain function and neurodegeneration 36, and cancer 37. Moreover, accumulating evidence suggests that miR‐9 is required for replication of multiple of viruses. Dong *et al*. 38 indicated a novel function of miR‐9 in influenza A virus infection and found that the influenza virus might hijack endogenous miR‐9 for the viral life cycle. Tatro *et al*. 39 suggested that HIV infection induced elevated expression of miR‐9, causing suppression of splice variants of KCNMA1, which may affect the release of neurotransmitters. Lai *et al*. reported that the nucleocapsid protein of human coronavirus OC43 causes activation of NFκB. This activation was the consequence of the nucleocapsid binding to RNA, specifically miR‐9 (a negative NFκB modulator), as was found in this study 40. Our study suggests that miR‐9 is a negative mediator for EV71 replication *in vitro* and *in vivo*. Ectopic expression of miR‐9 in cells resulted in inactivation of NFκB and ameliorated the excessive cytokine production, potentially lessening the organ injury induced by the cytokine storm during virus infection.

## Conclusions

Our data imply that antiviral activity of miR‐9 is related to regulation of the release of pro‐inflammatory cytokines through RIG‐I signal transduction via decreasing the activity and expression of NFκB. This study may provide new insights into EV71 infection suppression.

## Author contribution

In this work, BL and JZ conceived the study and designed the experiments, contributed to the data collection, performed the data analysis, and interpreted the results. BL wrote the manuscript and JZ contributed to the critical revision of article. Both authors read and approved the final manuscript.
